The article "Arabinose and xylose fermentation by recombinant Saccharomyces cerevisiae expressing a fungal pentose utilization pathway" was published in 2009. Journal: Microb Cell Fact.

# Arabinose and xylose fermentation by recombinant *Saccharomyces cerevisiae *expressing a fungal pentose utilization pathway

**DOI:** 10.1186/1475-2859-8-40

**Published:** 2009-07-24

**Authors:** Maurizio Bettiga, Oskar Bengtsson, Bärbel Hahn-Hägerdal, Marie F Gorwa-Grauslund

**Affiliations:** 1 Department of Applied Microbiology, Lund University, PO BOX 124, SE-22100 Lund, Sweden

## Abstract

**Background:**

Sustainable and economically viable manufacturing of bioethanol from lignocellulose raw material is dependent on the availability of a robust ethanol producing microorganism, able to ferment all sugars present in the feedstock, including the pentose sugars L-arabinose and D-xylose. *Saccharomyces cerevisiae *is a robust ethanol producer, but needs to be engineered to achieve pentose sugar fermentation.

**Results:**

A new recombinant *S. cerevisiae *strain expressing an improved fungal pathway for the utilization of L-arabinose and D-xylose was constructed and characterized. The new strain grew aerobically on L-arabinose and D-xylose as sole carbon sources. The activities of the enzymes constituting the pentose utilization pathway(s) and product formation during anaerobic mixed sugar fermentation were characterized.

**Conclusion:**

Pentose fermenting recombinant *S. cerevisiae *strains were obtained by the expression of a pentose utilization pathway of entirely fungal origin. During anaerobic fermentation the strain produced biomass and ethanol. L-arabitol yield was 0.48 g per gram of consumed pentose sugar, which is considerably less than previously reported for D-xylose reductase expressing strains co-fermenting L-arabinose and D-xylose, and the xylitol yield was 0.07 g per gram of consumed pentose sugar.

## Background

Bioethanol for transportation fuel can be produced in a sustainable way by fermentation of lignocellulosic raw materials, such as agricultural and forestry waste [1-3]. For the choice of the fermenting microorganism, complete substrate utilization, inhibitor tolerance and ethanol productivity are important aspects. The yeast *S. cerevisiae *satisfies the last two conditions [4-6], while metabolic engineering is required to obtain strains able to ferment L-arabinose and D-xylose, the most abundant pentose sugars in hemicellulose [6,7]. Although present in a smaller fraction than D-xylose, also L-arabinose needs to be efficiently converted to for overall process economy [8,9]. Furthermore, L-arabinose conversion to ethanol reduces carbon sources to be used by contaminant organisms competing with yeast.

*S. cerevisiae *strains able to ferment, in addition to hexose sugars, the pentose sugars L-arabinose and D-xylose have been obtained by heterologous expression of pathways of different origin [10,11]. Pentose sugars enter the pentose phosphate pathway (PPP) by conversion to D-xylulose (Figure 1) [12-20].

**Figure 1:** **Fungal L-arabinose and D-xylose utilization pathway**. AI: L-arabinose isomerase; ALX: L-xylulose reductase; AR: aldose reductase; LAD: L-arabitol dehydrogenase; R5PE: ribulose 5-phosphate epimerase; RK: ribulokinase; XDH: xylitol dehydrogenase; XI: D-xylose isomerase; XK: xylulokinase.

Bacteria convert L-arabinose to L-ribulose, L-ribulose-5-phosphate and finally D-xylulose-5-phosphate via L-arabinose isomerase (*araA*, EC 5.3.1.4) [16,21-23], L-ribulokinase (*araB*, EC 2.7.1.16) [14,21-23] and L-ribulose-5-P 4-epimerase (*araD*, EC 5.1.3.4) [14,15,21-23], respectively (Figure 1). D-xylose is directly isomerized to D-xylulose by D-xylose isomerase (*xylA*, EC 5.3.1.5) in bacteria and some anaerobic fungi [12,24,25].

In fungi, an aldose reductase (AR, EC 1.1.1.21) converts L-arabinose to L-arabitol and D-xylose to xylitol, respectively [18,26] (Figure 1). L-arabitol is converted by L-arabitol dehydrogenase (LAD, EC 1.1.1.12) [19,27] to L-xylulose, which is reduced to xylitol by L-xylulose reductase (ALX, EC 1.1.1.10) [19,28] (Figure 1). Thus, the L-arabinose pathway converges with the D-xylose pathway at the level of the achiral compound xylitol. Finally, xylitol is converted to D-xylulose by xylitol dehydrogenase (XDH, EC 1.1.1.9) (Figure 1) [29].

For the complete fermentation of the pentose fraction in lignocellulose hydrolyzate, a strain combining L-arabinose and D-xylose utilization is desired. Fermentation of either L-arabinose or D-xylose by recombinant *S. cerevisiae *has been demonstrated [10,11]. Co-fermentation of the two pentose sugars has been shown in strains expressing different pathway combinations. Co-fermenting laboratory and industrial *S. cerevisiae *strains have been obtained by combining the fungal reduction/oxidation D-xylose pathway with the bacterial isomerisation L-arabinose pathway [30,31]. More recently, a laboratory strain able to ferment both pentose sugars has been obtained by expressing D-xylose isomerase and the bacterial L-arabinose pathway and subsequent evolutionary engineering [32]. In strains expressing AR, conversion of L-arabinose to L-arabitol has been shown to be an unavoidable drawback, since L-arabitol inhibits the bacterial enzymes [30,31,33-35].

In the present work a new fungal pathway was reconstructed in a strain engineered for efficient for pentose fermentation [36]. The pathway combines *i) *an engineered mutant AR [37]; *ii) *a NAD^+^-dependent LAD from *Trichoderma reesei *(*Hypocrea jecorina*) [27]; *iii) *a NADH-dependent ALX from *Ambrosiozyma monospora *[28] and *iv) Pichia stipitis *XDH [38]. Strain TMB3043 (Table 1) was chosen as background since it has been endowed with genetic modifications allowing for improved pentose fermentation, such as overexpression of PPP [36] and XK [39] (Figure 1). In addition, TMB3043 harbors the deletion of *GRE3*, coding for an unspecific NADPH aldose reductase [40,41]. The removal of the Gre3p NADPH-dependent activity contributes to a more cofactor balanced pentose utilizing pathway.

**Table 1:** Plasmids and strains used in this study

**Plasmid**	**Features**	**Reference**
pUCsLAD1	pUC57 + synthetic sequence based on *T. reesei *Lad1p	Genscript Corp, Piscataway, USA

pUCsALX1	pUC57 + synthetic sequence based on *A. monospora *Alx1p	Genscript Corp, Piscataway, USA

YIpOB5	*ADH1p-XYL1*(K270R)-*ADH1t*, *PGK1p-XYL2-PGK1t*, *URA3*	[37]

YIpOB7	*TDH3p-ADH1t*, *PGK1p-XYL2-PGK1t*, *URA3*	Bengtsson O, Bettiga M, Garcia-Sanchez R, Gorwa-Grauslund MF: **Differential behaviour of two commonly used promoters in xylose utilizing recombinant *Saccharomyces cerevisiae; ***unpublished.

YIpOB9	*TDH3p-XYL1*(K270R)-*ADH1t*, *PGK1p-XYL2-PGK1t*, *URA3*	This work

p425GPD	*TDH3*p-*CYC1*t, *LEU2*	[44]

p425GPD_LAD1	*TDH3*p-*lad1*(*T. reesei*, cDNA)- *CYC1*t, *LEU2*	This work

p425GPD_ALX1	*TDH3*p-*ALX1*(*A. monospora*)- *CYC1*t, *LEU2*	This work

p425GPD_sLAD1	*TDH3*p-*sLAD1*(synthetic)- *CYC1*t, *LEU2*	This work

p425GPD_sALX1	*TDH3*p-*sALX1*(synthetic)- *CYC1*t, *LEU2*	This work

p425GPD_sLAD1_sALX1	*TDH3*p-*sLAD1*(synthetic)- *CYC1*t; *TDH3*p-*sALX1*(synthetic)- *CYC1*t, *LEU2*	This work

**Strain**	**Genotype**	**Reference**

*T. reesei *Rut-C30	Wild type	NRRL 11460

*A. monospora *PYCC4390^T^	Wild type	Kindly provided by Prof. Isabel Spencer-Martins

CEN.PK 113-16B	*MAT*a, *leu2-3 112*	[47]

TMB3043	CEN.PK 2-1C, *MAT*a, *leu2-3 112, ura3-52*, *Δgre3*, *his3::HIS3 PGK1p-XKS1-PGK1t*, *TAL1::PGK1p-TAL1-PGK1t*, *TKL1::PGK1p-TKL1-PGK1t*, *RKI1::PGK1p-RKI1-PGK1t*, *RPE1::PGK1p-RPE1-PGK1t*	[36]

TMB3656	CEN.PK 113-16B, p425GPD_ALX1	This work

TMB3657	CEN.PK 113-16B, p425GPD_LAD1	This work

TMB3658	CEN.PK 113-16B, p425GPD_sALX1	This work

TMB3659	CEN.PK 113-16B, p425GPD_sLAD1	This work

TMB3660	CEN.PK 113-16B, p425GPD	This work

TMB3662	TMB3043, YIpOB9	This work

TMB3664	TMB3662, p425GPD_sLAD1_sALX1	This work

TMB3665	TMB3662, p425GPD	This work

The AR encoded by the mutated *P. stipitis XYL1*(K270R) has been engineered for an increased NADH preference compared with the natural enzyme [37,42,43]. Expression of the mutated gene allowed a more coenzyme-balanced D-xylose utilization, with increased D-xylose utilization rate and reduced xylitol formation when integrated in a single copy [37].

## Results

### Reconstruction of an improved fungal pentose utilization pathway in *S. cerevisiae*

TMB3043 was transformed with mutated *XYL1*(K270R), coding for aldose reductase (AR) and *XYL2*, coding for xylitol dehydrogenase (XDH), both inserted in the integrative plasmid YIpOB9 (Table 1), and the new strain was named TMB3662 (Table 1). The complete pentose utilizing pathway was introduced in *S. cerevisiae *by transforming TMB3662, carrying integrated AR and XDH, with the multicopy plasmid harboring the synthetic, codon optimized genes *sLAD1 *and *sALX1*, coding for L-arabitol dehydrogenase (LAD) and L-xylulose dehydrogenase (ALX), respectively (Table 1). This strain, containing a complete L-arabinose pathway, consisting of AR, LAD, ALX and XDH was named TMB3664. In addition, a D-xylose-only utilizing strain was constructed by transforming TMB3662 with plasmid p425GPD, [44] lacking the structural genes coding for LAD and ALX (Table 1). This strain, containing only AR and XDH, was named TMB3665 (Table 1).

### Enzyme activities

The successful expression of the pentose metabolizing enzymes was verified by measuring the individual enzyme activities. The results are summarized in Table 2 and 3. Table 2 includes enzyme activity values for the reductases AR and ALX. Table 3 includes enzyme activity values for the dehydrogenases LAD and XDH, as well as an activity referred to as "polyol dehydrogenase", combining LAD, XDH and ALX. In fact, when LAD and XDH enzymes are co-present, NAD^+ ^reduction coupled with L-arabitol oxidation could be the result of the combined activity of LAD and XDH (Figure 1). In addition, in strains where LAD, ALX and XDH are co-expressed, a further contribution is given by ALX activity with NAD^+ ^as a cofactor when xylitol is the substrate (Figure 1, Table 3). For this reason L-arabitol and xylitol oxidizing activity with NAD^+ ^as cofactor is referred to as "polyol dehydrogenase" [45].

**Table 2:** Enzyme activities (U/(mg total protein)): reductases

**Enzyme**	**Substrate**		**Strain**
AR	D-XYLOSE	L-ARABINOSE	
	
	0.70 ± 0.04	0.82 ± 0.01	TMB3662
	
	0.47 ± 0.05	0.53 ± 0.03	TMB3664
	
	0.67 ± 0.03	0.80 ± 0.07	TMB3665

ALX^b^	XYLITOL^a^	L-ARABITOL^a^	
	
	11.20 ± 1.40	0.00	TMB3658

ALX	L-XYLULOSE		
	
	3.01 ± 0.50		TMB3664
	
	0.00		TMB3665

b. NAD^+ ^as a cofactor (reverse reaction). NADH was used as a cofactor for all other reactions.

**Table 3:** Enzyme activities (U/(mg total protein)): dehydrogenases

**Enzyme**	**Substrate^a^**		**Strain**
LAD	L-ARABITOL	XYLITOL	
	
	0.77 ± 0.10	0.58 ± 0.07	TMB3659

ALX^a^, LAD, XDH	0.94 ± 0.04 (0.45 ± 0.02)	28.54 ± 4.91 (21.13 ± 5.57)	TMB3664

XDH	0.72 ± 0.01 (0.25 ± 0.00)	7.20 ± 0.56 (7.88 ± 0.88)	TMB3665

NAD^+ ^was used as a cofactor for all reactions. a. Standard substrate concentration: 330 mM. Values between parentheses are referred to assays performed with substrate concentration of 100 mM.

First, AR activity of the mutant AR(K270R) with L-arabinose as substrate and NADH as cofactor was verified using cell extracts from TMB3662. The mutated AR(K270R) enzyme retained its catalytic activity with L-arabinose as substrate, with a specific activity of 0.82 ± 0.01 U/(mg total protein), compared with 0.70 ± 0.04 U/(mg total protein) when D-xylose was used as substrate (Table 2). The slightly higher reductase activity for L-arabinose is consistent with previously reported data for the natural enzyme [46].

Next, active expression of the codon optimized *sLAD1 *and *sALX1 *in *S. cerevisiae *was verified by measuring LAD activity and ALX activity (Table 2 and 3) in cell extracts from strains expressing these enzymes alone (TMB3659 and TMB3658, respectively, Table 1). LAD and ALX activity was also measured in cell extracts from analogous strains, expressing the natural *lad1 *and *ALX1 *genes individually in the same genetic background (TMB3657 and TMB3656, respectively, Table 1). The enzymatic activities were not significantly different, indicating that in this case codon optimization did not influence enzymatic activity (data not shown). Nevertheless, the synthetic gene versions were chosen for the continued work.

The LAD activity was 0.77 ± 0.1 U/(mg total protein) with L-arabitol as a substrate and 0.58 ± 0.07 U/(mg total protein) with xylitol (Table 3). The ALX activity was measured with NAD^+ ^as cofactor (reverse reaction, see Methods section). The activity was 11.2 ± 1.4 U/(mg total protein) when xylitol was used as a substrate, while no activity was detected with L-arabitol (Table 2), in agreement with previous reports [28,45]. No significant activity (< 0.05 U/(mg total protein)) with either substrate was detected in the original host strain CEN.PK 113-16B [47] (data not shown).

Finally, all heterologous activities introduced in strains TMB3664, expressing AR, LAD, ALX and XDH and TMB3665, expressing AR and XDH, were measured. The AR activity in strain TMB3665 was essentially identical to that of the parental strain TMB3662 (Table 2), while the AR activity for TMB3664 was only about 65% of the parental strain. This could be due to lower expression owing to the metabolic burden of expressing two additional genes on a multicopy plasmid. Alternatively, L-arabitol and xylitol formed in the *in vitro *reaction could be re-oxidized by LAD and ALX, regenerating NADH and thus reducing the apparent activity of AR in cell extracts of TMB3664 (Figure 1). The difference in enzyme activity did, however, not influence D-xylose utilization (See below and Table 4).

**Table 4:** Substrate consumption and product formation parameters during anaerobic batch fermentation of mixed sugars in defined mineral medium

		**TMB3664** **(D-xylose/L-arabinose pathway)**		**TMB3665** **(D-xylose pathway)**
	
	**Medium**	G-A-X	G-A	G-A-X
**Overall process**	Initial glucose g/l	20.7 ± 0.2	20.1 ± 0.9	20.1 ± 0.4
	
	Initial L-arabinose g/l	22.1 ± 0.2	23.1 ± 0.4	22.1 ± 0.1
	
	Initial xylose g/l	21.7 ± 0.4	-	20.8 ± 0.3
	
	Consumed arabinose g/l	3.9 ± 0.2	2.1 ± 0.1	3.1 ± 0.3
	
	Consumed xylose g/l	14.1 ± 0.2	-	13.7 ± 0.2
	
	Final ethanol titer^+^ g/l	15.3 ± 0.0	9.3 ± 0.4	14.3 ± 0.3
	
	Y ethanol, total sugars (g ethanol)/(g sugar)	0.23 ± 0.00	0.21 ± 0.01	0.22 ± 0.01
	
	Y ethanol, consumed sugars (g ethanol)/(g sugar)	0.40 ± 0.01	0.42 ± 0.01	0.39 ± 0.00
	
	Y xylitol, consumed xylose (g xylitol)/(g consumed D-xylose)	0.09 ± 0.01	-	0.10 ± 0.0
	
	Y xylitol, consumed C5 (g xylitol) (g consumed sugar)^-1^	0.07 ± 0.00	n.d.	0.08 ± 0.0
	
	Y arabitol, consumed arabinose (g L-arabitol)/(g consumed L-arabinose)	0.48 ± 0.01	0.39 ± 0.03	0.90 ± 0.07

				

Pentose Phase^a^	q arabinose (g L-arabinose)/(g cells)/h	0.021 ± 0.001	0.011 ± 0.001	0.013 ± 0.000
	
	q xylose (g D-xylose)/(g cells)/h	0.080 ± 0.001	-	0.077 ± 0.001
	
	q ethanol (g ethanol)/(g cells)/h	0.035 ± 0.001	0.003 ± 0.001	0.029 ± 0.001
	
	Biomass, produced from C5 g/l	0.37 ± 0.01	n.d.	0.25 ± 0.03
	
	Y biomass, produced from C5 (g biomass)/(g consumed sugar)	0.025 ± 0.001	-	0.019 ± 0.002
	
	Y ethanol, produced from C5 (g ethanol)/(g consumed sugar)	0.35 ± 0.01	0.35 ± 0.01	0.32 ± 0.01
	
	Y glycerol, produced from C5 (g glycerol)/(g sugar)	0.03 ± 0.01	0.06 ± 0.02	0.02 ± 0.00

Values are the calculated average of two biological replicates. Errors are given as mean deviations. G-A-X: medium containing glucose, L-arabinose and D-xylose; G-A: medium containing glucose and L-arabinose only. +: estimated based on the degree of reduction balance. a. values calculated after glucose depletion. q: specific productivity, Y: yield, C5: pentose sugar, n.d.: not detected.

ALX specific activity was 3.01 U/(mg total protein) in TMB3664 and not detectable in TMB3665 (Table 2). In the presence of NADH, XDH can act as a D-xylulose reductase[38], while no report on L-xylulose conversion by XDH is available. However, the absence of ALX activity in TMB3665 may indicate that this enzyme does not accept the L-xylulose stereoisomer as substrate, although a specific assay would be needed to confirm this speculation.

The polyol dehydrogenase activity was measured in strains TMB3664 and TMB3665 using L-arabitol and xylitol at different concentrations (Table 3). Consistent with the expression of *sLAD1 *in TMB3664, the dehydrogenase activity whith L-arabitol as a substrate was higher in this strain than in TMB3665. The activity difference increased when L-arabitol, a preferred substrate for LAD but not for XDH [27,38,45], was used at a concentration of 100 mM instead of 330 mM (Table 3). The ratio between the activity in TMB3665 and TMB3664 was ~0.75 at 330 mM and ~0.55 at 100 mM, respectively (Table 3) [28]. The co-existence of LAD, ALX and XDH activities in TMB3664 conferred three to four times higher xylitol dehydrogenase activity, 28.54 U/(mg total protein), compared with 7.2 U/(mg total protein) for TMB3665 (Table 3). Thus, the recombinant *S. cerevisiae *strain TMB3664 harbors enzymatic activities for L-arabinose and D-xylose utilization comparable to those previously measured in natural yeast species capable of fast pentose sugar consumption [45].

### Growth on pentose sugars

The ability of the recombinant *S. cerevisiae *strain TMB3664 to utilize L-arabinose and D-xylose as sole carbon source for growth was first assessed in aerobic culture in mineral media containing either of the pentose sugars as sole carbon source. TMB3664 was able to utilize both pentose sugars for growth. The maximum specific growth rate was 0.05 ± 0.003 h^-1 ^and 0.05 ± 0.002 h^-1 ^in L-arabinose and D-xylose medium, respectively. With L-arabinose, the strain reached a final cellular density, expressed as OD_620 nm_, of 11.2 ± 0.6 after ~100 h. The final OD in D-xylose medium was 18.7 ± 0.9 and it was reached in 90 h. No growth was detected after more than 5 days in L-arabinose medium for the control strain TMB3665, while in D-xylose medium the growth rate 0.06 ± 0.002 h^-1^, and final OD, 19.1 ± 0.8, were similar to TMB3664.

### Anaerobic mixed sugar fermentation

The anaerobic fermentation capacity of the L-arabinose and D-xylose utilizing strain TMB3664 was assessed in batch culture with a mixture of glucose, L-arabinose and D-xylose as a carbon source (Figure 2 and Table 4).

**Figure 2:** **Substrate and product concentration during anaerobic batch fermentation of defined mineral medium containing glucose, L-arabinose and D-xylose**. (A) L-arabinose and D-xylose utilizing strain TMB3664; (B) D-xylose utilizing strain TMB3665. Primary (left) Y axis: filled circles: glucose; filled squares: D-xylose; filled triangles: L-arabinose; filled diamonds: ethanol; empty circles: glycerol. Secondary (right) Y axis: empty squares: xylitol; empty triangles: L-arabitol; stars: dry cell weight. The figure illustrates one representative batch of duplicate experiments for each strain.

Glucose was utilized first and completely consumed after 30 hours (Figure 2). A minor fraction of pentose sugars was co-consumed with glucose; nonetheless L-arabinose and D-xylose consumption rates were higher after glucose depletion in the subsequent pentose fermentation phase. The specific growth rate during initial growth on glucose was μ = 0.109 ± 0.003 h^-1^. Biomass formation continued in the pentose fermentation phase. It was, however, not possible to calculate the specific growth rate, although the biomass concentration increased reproducibly from ~1.4 g/l at the point of glucose depletion to ~1.8 g/l at the end of the fermentation. Specific substrate consumption and product formation rates (Table 4) were calculated only for the pentose phase, as described in the Materials and Methods section.

Besides ~20 g/l of glucose, the strain consumed 3.9 g/l of L-arabinose and 14.1 g/l of D-xylose. The consumption rate after glucose depletion was 0.020 g/(g cells)/h for L-arabinose and 0.080 g/(g cells)/h for D-xylose. Produced ethanol was in total 15.3 g/l (estimated based on the degree of reduction balance [48]), with a specific productivity from pentose sugars of 0.035 g/(g cells)/h. Ethanol yield was 0.23 g/(g sugar) based on total sugars present at the beginning of the fermentation, 0.40 g/(g sugar) based on consumed sugars and 0.35 g/(g sugar) based on consumed pentose sugars, as calculated after glucose depletion.

The L-arabitol yield for TMB3664 was 0.48 g/(g consumed L-arabinose) demonstrating for the first time in an AR expressing strain, that L-arabinose was not only converted to L-arabitol [30,31,49], but further channeled into the metabolism. The xylitol yield was only 0.09 g/(g consumed D-xylose), comparable to previously reported yield obtained with strains expressing mutant AR with increased preference for NADH [37,42,43,50].

Fermentation with an identical set up was performed with the control strain TMB3665 (Table 1), in order to evaluate the advantage given to TMB3664 by capacity of metabolizing L-arabinose (Table 4). As shown in Figure 2, the overall behavior of the strain was similar to strain TMB3664. However, L-arabinose was taken up at a slower rate of 0.013 g/(g cells)/h and almost entirely excreted as L-arabitol (Table 4). The ethanol yield calculated on total consumed sugars was 0.39 g/(g sugar). Biomass and glycerol yields from to the pentose phase (Table 4) were slightly but reproducibly higher in the L-arabinose consuming strain TMB3664 than in the control strain TMB3665 (Table 4). In addition, the xylitol yield was about 10% higher in TMB3665, which could be ascribed to the unspecific substrate preference of LAD present in TMB3664 [27].

Finally, anaerobic fermentation was performed with TMB3664 in batch containing only glucose and L-arabinose as a carbon source (Table 4). In this setup, cells grew anaerobically on glucose at μ = 0.113 ± 0.06 h^-1^, co-consuming a small amount of L-arabinose. Biomass formation ceased after glucose depletion and no anaerobic growth was observed in the L-arabinose phase. Cells continued to consume L-arabinose at a rate of 0.011 g/(g cells)/h until the end of the fermentation at t = 120 hours (Table 4). The final ethanol concentration (estimated based on the degree of reduction balance [48]) was 9.3 g/l, with a yield of 0.21 g/(g sugar) based on total sugars present at the beginning of the fermentation, 0.42 g/(g sugar) based on consumed sugars and 0.35 g/(g sugar) based on consumed L-arabinose (Table 4). By-product yields were lower than when D-xylose was also present in the medium. In fact, the xylitol concentration was below the detection limit and the L-arabitol yield was 0.39 g/(g of consumed L-arabinose) (Table 4).

## Discussion

The investigation presented herein aimed at constructing and characterizing a recombinant *S. cerevisiae *strain with enhanced capacity to ferment mixtures of glucose and pentose sugars. The strain harbored and improved fungal pathway for arabinose and xylose utilization. In fact, in anaerobic conditions the strain fermented both L-arabinose and D-xylose. This was not the first time that a recombinant *S. cerevisiae *harboring a fungal pentose utilization pathway was obtained [51]. However, the present report shows an improvement of more than one order of magnitude in L-arabinose utilization when compared to previous similar attempts [51]. Consistently, the aerobic growth rate on L-arabinose as sole carbon source also showed an estimated 10 fold increase [52].

The currently best L-arabinose fermenting *S. cerevisiae *strains have been obtained by expression of the bacterial L-arabinose pathway alone [53] (Figure 1), or in combination with a D-xylose isomerase pathway (Figure 1) [32,54]. For these constructs, co-fermentation of the two pentose sugars has only been achieved by extensive and carefully controlled evolutionary engineering protocols [32]. In particular, it was demonstrated that evolutionary engineering of combined traits such as fermentation of two sugars easily drifts towards one of the traits, as soon as it becomes preferred over the other. In a mixture of D-xylose and L-arabinose, the selection process towards the utilization of D-xylose accelerated as soon as a preference for D-xylose arose, to the disadvantage of L-arabinose utilization. Thus, co-fermentation of L-arabinose and D-xylose was the result of a delicate equilibrium of different selection pressures, with a yet un-clarified molecular explanation.

In contrast, the present study showed that the presence in TMB3664 of the additional activities needed for L-arabinose fermentation did not affect D-xylose fermentation at all. At the rates observed in the current study, arabinose fermentation rather improved ethanolic fermentation of D-xylose, indeed representing a pure net advantage for the strain in sugars mixtures (Table 4).

L-arabinose and D-xylose co-utilization by *S. cerevisiae *has previously been demonstrated by combining a bacterial L-arabinose isomerase pathway and a fungal reduction/oxidation D-xylose pathway [30,31] (Figure 1). However, AR expressing strains convert L-arabinose to L-arabitol [30,31], which represents a dead end in the metabolism of such strains and, in addition, can inhibit the bacterial enzymes for L-arabinose utilization [30,31,33-35]. Thus, a solution to this problem was to exploit the natural efficiency of AR to convert L-arabinose to L-arabitol, and to further channel L-arabitol into central metabolism via the fungal L-arabinose utilizing pathway (Figure 1). Therefore, strain TMB3664 was constructed by expressing an improved fungal pentose utilization pathway, combining a mutated AR engineered for enhanced NADH preference with strictly NAD^+^/NADH dependent ALX, LAD and XDH. Indeed, more than 50% of the L-arabitol generated by AR in strain TMB3664 was further channeled into central metabolism in anaerobic mixed sugar fermentation. In addition, the yield of the second by-product xylitol was reduced to less than 10%.

The enzymes involved in the reduction-oxidation steps of fungal pentose sugar assimilation display different co-factor preferences [45]. By-product accumulation [55], poor aerobic growth [52] and poor anaerobic ethanol production [51] not only in recombinant *S. cerevisiae *strains, but also in natural L-arabinose consuming yeast species such as *Candida arabinofermentans *and *P. guilliermondii*, have been ascribed to the difference in co-factor preference of the L-arabinose metabolizing enzymes [45,56]. The activity of the heterologous enzymes expressed in *S. cerevisiae *TMB3664 was 5 to 50 times higher than previously reported for similarly constructed recombinant *S. cerevisiae *strains [28,52] and comparable to the enzyme activity levels found in natural L-arabinose fermenting yeast [45]. The pathway reconstructed in TMB3664 combines a mutant AR, with increased relative coenzyme preference for NADH [37], with an entirely NAD^+^/NADH dependent downstream pathway [27,28,38]. This partially relieved the strain from NAD^+ ^regeneration [45,56] and allowed it to channel L-arabinose and D-xylose towards the formation of ethanol and even biomass, with reduced by-product formation.

L-arabinose metabolism of the natural pentose fermenting yeasts *C. arabinofermentans *and *P. guilliermondii *has been characterized in relation to sugar concentration and aeration [56]. Although these yeast strains were not grown under strict anaerobic conditions, it may still be useful to compare the product formation pattern of TMB3664 with those of *C. arabinofermentans *and *P. guilliermondii *grown in different aeration conditions including severe oxygen limitation [56]. *C. arabinofermentans *consistently produced less L-arabitol than *P. guilliermondii*, except under the most extreme oxygen limitation, when both yeast strains displayed an L-arabitol yield on consumed L-arabinose of approximately 0.6 g/g. Considering that, in contrast to *P. guilliermondii, C. arabinofermentans *exhibits moderate but detectable NADH-dependent ALX activity, in addition to high NAD^+^-dependent LAD activity [45], it is tempting to rank the three yeast strains in terms of co-factor balance of their pentose utilization pathway and to relate this to the strains' L-arabitol and xylitol formation. Thus, TMB3664, harboring the mutated AR and the exclusively NADH-dependent ALX from *A. monospora*, would be considered the most co-factor balanced of the three strains, and in fact it produces the lowest yield of L-arabitol and xylitol and has the highest ethanol production rate [45,56]. This comparison delineates a trend and points out the importance of equilibrated co-factor utilization for minimal by-product formation in pentose fermenting recombinant *S. cerevisiae *strain based on a reduction/oxidation pathway for pentose metabolism.

In conclusion, the present work describes an L-arabinose and D-xylose co-fermenting recombinant *S. cerevisiae *strain expressing a pentose utilization pathway of entirely fungal origin. Anaerobic product formation by such strains such strains is largely influenced by the co-factor preference of the enzymes constituting the pathway.

## Materials and methods

### Strains and media

Microbial strains and plasmids utilized for this work are summarized in Table 1. *Escherichia coli DH5a *(Life Technologies, Rockville, USA) was used as intermediate host for cloning steps and plasmid amplification and was routinely grown in LB medium [57] containing 100 mg/l ampicillin (Shelton scientific, Shelton, USA). *S. cerevisiae *strains were grown aerobically in Yeast Nitrogen Base medium (YNB, Difco Laboratories-Becton, Dickinson & Co., Sparks, USA), buffered at pH 5.5 with 50 mM potassium hydrogen phthalate (Merck, Darmstadt, Germany) [58] and formulated as it follows; YNBG: 20 g/l glucose, 6.7 g/l YNB; YNBA: 50 g/l L-arabinose, 13.4 g/l YNB; YNBX: 50 g/l D-xylose, 13.4 g/l YNB. According to strain requirements, the medium was supplemented with uracil and/or leucine at concentrations of 40 mg/l and 240 mg/l, respectively. Solid media were obtained by addition of 20 g/l agar (Merck, Darmstadt, Germany). Anaerobic mixed sugar batch fermentation was performed in defined mineral medium [50] supplemented with 0.4 g/l Tween 80 (Sigma-Aldrich, St. Louis, USA), 0.01 g/l ergosterol (Alfa Aesar, Karlsruhe, Germany), glucose (VWR International, Poole, UK), D-xylose (Acros Organics, Geel, Belgium) and L-arabinose (Sigma-Aldrich, St. Louis, USA) each at the concentration of 20 g/l or glucose and L-arabinose, each at the concentration of 20 g/l.

### Nucleic acid manipulation

Standard molecular biology techniques were used [57]. *T. reesei *and *A. monospora *chromosomal DNA was extracted using a bead-beater (Biospecs products, Bartlesville, OK, USA) and phenol/chloroform [57].

Plasmid DNA was purified from *E. coli *with Gene JET plasmid miniprep kit (Fermentas, Vilnius, Lithuania). Agarose gel DNA extractions were made using the QIAquick^® ^Gel Extraction Kit (Qiagen GmbH, Hilden, Germany). Purification of PCR products was made with the E.Z.N.A.^® ^Cycle-Pure Kit (Omega Bio-tek Inc, Doraville, GA, USA). Primers for PCR and sequencing service were purchased from Eurofins MWG Operon (Ebersberg, Germany). DNA modifying enzymes, restriction endonucleases and polymerases were purchased from Fermentas, Vilnius, Lithuania. Gene synthesis service was purchased from Genscript corp. (Piscataway, USA). Analytical PCR was performed with Taq DNA polymerase while preparative PCR was performed with High Fidelity PCR Enzyme Mix. Calf intestinal alkaline phosphatase and T4 DNA Ligase were used for DNA dephosphorylation and ligation, respectively. The lithium acetate/dimethyl sulfoxide protocol was used for yeast transformation [59].

### Gene cloning and plasmid construction

The *XYL1*(K270R) gene fragment was excised from plasmid YIpOB5 [37] and inserted into YIpOB7 [Bengtsson O, Bettiga M, Garcia-Sanchez R, Gorwa-Grauslund MF: **Differential behaviour of two commonly used promoters in xylose utilizing recombinant *Saccharomyces cerevisiae***, unpublished] using the *XbaI *restriction sites, creating plasmid YIpOB9 (Table 1). The constructed plasmid was analyzed with restriction analysis and PCR to confirm correct insertion. The inserted part was sequenced to verify that no mutations were introduced.

The *T. reesei *(*H. jecorina*) gene *lad1 *codes for a NAD^+^-dependent L-arabitol dehydrogenase [27], while *A. monospora ALX1 *codes for a NADH-dependent L-xylulose reductase [28,45] (Figure 1). *T. reesei lad1 *contains an intron of 69 base pairs [27]. First, the two exons were separately PCR amplified using *T. reesei *chromosomal DNA as template. Exon N.1 was PCR amplified with primers containing the restriction site *BamHI *(LAD-BamHI-FW: 5'-TAGA***GGATCC***ATGTCGCCTTCCGCAGTCGATGAC) and a 24-base region overlapping exon N.2 (LAD-Ex1-R: 5'-***GGACATCTGAACCACAGATACC***AGTGCTGCGGAC). Exon N.2 was PCR amplified with primers containing a 24-base region overlapping exon N.1 (LAD-Ex2-F: 5'-***CTGGTATCTGTGGTTCAGATGTCC***ATTTCTGGCACG) and the restriction site *HindIII *(LAD-HindIII-RV: 5'-CAGC***AAGCTT***TCTAGATCAATCCAGGCTCTGAATCATG). The two PCR products were purified and pooled in a new PCR reaction, carried out with primers LAD-BamHI-FW and LAD-HindIII-RV and yielding the complete coding sequence of *lad1*. The PCR product was inserted into the vector p425GPD [44] creating the plasmid p425GPD_LAD1 (Table 1).

*ALX1 *was PCR-amplified using *A. monospora *chromosomal DNA as template with primers containing the restriction sites for *SpeI *(ALX-SpeI-FW: 5'-GCT***ACTAGT***AGATCTATGACTGACTACATTCCAACTT) and *XhoI *(ALX-Xho-RV: 5'-TTA***CTCGAG***AGATCTTTACCAAGAAGTGAAACCACCAT). The PCR product was inserted into the vector p425GPD [44] creating plasmid p425GPD_ALX1 (Table 1).

Based on the published amino acid sequence of Lad1p and Alx1p (Genebank accession numbers AF355628 and AJ583159, respectively), the corresponding optimized DNA sequences were synthesized and the synthetic genes were designated *sLAD1 *and *sALX1*, respectively. Synthetic sequences were designed taking into account *S. cerevisiae *codon usage and the possible presence of secondary structure generating sequences, according to a proprietary algorithm of Genscript Corp (Genscript Corp., Piscataway, USA). A fragment containing *sLAD1 *was excised from the vector pUCsLAD1 (Table 1) by digestion with *BamHI *and *HindIII *and inserted into the vector p425GPD [44] creating plasmid p425GPD_sLAD1 (Table 1). A fragment containing *sALX1 *was excised from the vector pUCsALX1 (Table 1) by digestion with *SpeI *and *XhoI *and inserted into the vector p425GPD [44] creating plasmid p425GPD_sALX1 (Table 1). The cassette consisting of *TDH3 *promoter, *sALX1 *and *CYC1 *terminator was PCR-amplified from plasmid p425GPD_sALX1 with primers containing the restriction site *SapI *(Cass-Sap-FV: 5'-***GCTCTTCCGCTT***GGTACCGGCCGCAAATTAAAG and Cass-Sap-RV: 5'-***AAGCGGAAGAG***CCAGTTTATCATTATCAATACTCGCC). The PCR product was inserted into plasmid p425GPD_sLAD1 creating plasmid p425GPD_sLAD1_sALX1 (Table 1). Each new construct was sequenced to verify the absence of mutations.

### Cultivation conditions

*S. cerevisiae *was grown aerobically in Erlenmeyer baffled flasks filled to maximum 1/10 of the volume with medium, incubated at 30°C in a rotary shake-incubator (INR-200 shake incubator, Gallenkamp, Leicester, UK) at 200 rpm. Cultures were inoculated at an initial O.D._620 nm _of 0.20 ± 0.02 with sterile H_2_O-washed cells from a late-exponential YNBG pre-culture. The maximum specific growth rate, μ, was calculated from exponential fitting of growth curves from at least two biological duplicates. Anaerobic mixed-sugar batch fermentation was performed in 1.5 l working volume bioreactors (Sartorius Stedim Biotech S.A., Aubagne, France), for 120 h, at 30°C, 200 rpm and at pH 5.5 automatically controlled by addition of 3 M KOH. Anaerobic conditions were established prior to inoculation by sparging the medium for at least 3 hours with nitrogen gas (< 5 ppm O_2_, AGA, Malmö, Sweden) at 0.2 l/min flow rate. A water-lock was placed at the fermentor gas outlet. Cells were pre-grown aerobically in shake flasks in defined mineral medium [50], harvested by centrifugation, resuspended in ~10 ml sterile medium and inoculated into the fermentor at an initial O.D._620 nm _of 0.20 ± 0.02. Fermentation experiments were performed in duplicate.

### Enzyme activity

For crude protein extract preparation, cells were grown in 100 ml YNBG medium until O.D._620 nm _of 1, harvested and stored at -80°C. Proteins were extracted with Yeast Protein Extraction Reagent (YPER, Pierce, Rockford, IL, USA) according to the manufacturer's instructions. Protein concentration was determined with Coomassie Protein Assay Reagent (Pierce, Rockford, IL, USA). All activity measurements were performed on fresh extracts. Aldose reductase activity [46,60] was measured essentially as previously described. Where indicated, L-arabinose was used as a substrate instead of D-xylose. L-arabitol dehydrogenase activity [20,38] was measured as previously described. L-xylulose reductase [28], xylitol dehydrogenase [38] and global polyol dehydrogenase activities were measured as previously described. Where indicated, a substrate concentration of 100 mM instead of 330 mM and L-arabitol instead of xylitol were used. Only NAD^+ ^and NADH were used as cofactors. Enzyme activity measurements were performed in triplicate at least on extracts from two independent cultivations. For all the activities measured, 1 U is defined as the amount of enzyme converting 1 μmol of substrate per minute in the conditions of the assay.

### Analyzes

Samples were drawn from the fermentors after discharging the sample tubing dead-volume, cells were separated by centrifugation and the supernatant was filtered through 0.20 μm membrane filters (Toyo Roshi Kaish, Tokyo, Japan) and stored at 4°C until further analysis.

Concentration of glucose, D-xylose, acetate and glycerol and ethanol was determined by HPLC (Beckman Instruments, Fullerton, USA). The compounds were separated with three Aminex HPX-87H resin-based columns (Bio-Rad, Hercules, USA) connected in series and preceded by a Micro-Guard Cation-H guard column (Bio-Rad, Hercules, USA). Separation was performed at 45°C, with 5 mM H_2_SO_4 _at a flow rate of 0.6 ml/min as mobile phase. Concentration of L-arabinose, L-arabitol and xylitol was determined by HPLC (Waters, Milford, USA) using two HPX-87P resin-based column (Bio-Rad, Hercules, USA) preceded by a Micro-Guard Carbo-P guard column (Bio-Rad, Hercules, USA). Separation was performed at 80°C, with H_2_O at a flow rate of 0.5 ml/min as mobile phase. All compounds were quantified by refractive index detection (Shimadzu, Kyoto, Japan). For each HPLC run, a 7-point calibration curve was made for each compound to calculate concentrations. Each sample was analyzed at least in duplicate and a maximum of 10% difference between replicate analyzes was accepted.

For each fermentation experiment, cell dry weight was determined at least in three points, in triplicate for each point. The end point of the fermentation (t = 120 h) was always included. For dry weight determination, a known volume of cell culture was filtered through dry pre-weighed 0.45 μm nitrocellulose filters, which were subsequently dried in a microwave oven and weighed. Because of evaporation, ethanol concentration was calculated from the degree of reduction balance of the overall carbon stoichiometry of the fermentation [48]. Evaporated ethanol was always <10% of the total ethanol present at the end of the fermentation. Substrate consumption and product formation rates during the pentose phase (Table 4) were calculated as average rates. Total consumed D-xylose and L-arabinose and average biomass concentration between the point of glucose depletion and the end of the fermentation were used for the calculation.

## Abbreviations

AR: aldose reductase; ALX: L-xylulose reductase; HPLC: high performance liquid chromatography; LAD: L-arabitol dehydrogenase; NADH: nicotinamide adenine dinucleotide; NADPH: nicotinamide adenine dinucleotide phosphate; OD: optical density; PCR: polymerase chain reaction; PPP: pentose phosphate pathway; XDH: xylitol dehydrogenase; XI: D-xylose isomerase; XK: xylulokinase; XR: D-xylose reductase; YNB: yeast nitrogen base; YNBA: yeast nitrogen base/L-arabinose; YNBG: yeast nitrogen base/glucose; YNBX: yeast nitrogen base/D-xylose.

## Competing interests

The authors declare that they have no competing interests.

## Authors' contributions

MB participated in the design of the study, performed the experimental work and wrote the manuscript. OB performed the experimental work. BHH participated in the design of the study and commented on the manuscript. MFGG participated in the design of the study and commented on the manuscript. All the authors read and approved the final manuscript.
